# Diagnostic Accuracy of Procalcitonin for Bacterial Infection in Liver Failure: A Meta-Analysis

This article has been retracted.

**DOI:** 10.1155/2021/5801139

**Published:** 2021-07-05

**Authors:** Xinchun He, Liang Chen, Haiou Chen, Yuqing Feng, Baining Zhu, Caixia Yang

**Affiliations:** Department of Infectious Disease, Hunan Provincial People's Hospital (The First Affiliated Hospital of Hunan Normal University), Changsha, Hunan 410005, China

## Abstract

The purpose of our studies was to systematically assess the accuracy and clinical value of plasma calcitonin in patients with liver failure complicated with bacterial infection. In this study, we included prospective observational studies or randomized controlled trials on PCT. The quality of the studies was evaluated using the Quality Assessment of Diagnostic Accuracy Studies-2 (QUADAS-2) tool. Heterogeneity, pooled diagnostic odds ratio (DOR), pooled sensitivity, pooled specificity, pooled positive likelihood ratio, pooled negative likelihood ratio, the area under the summary receiver operating characteristic curve (SROC), and metaregression analysis were performed using Stata16.0 software. Consequently, the studies revealed substantial heterogeneity (*I*^2^ = 96, 95% confidence interval (95% CI) = 94–99). The results of meta-analysis using random effect models suggested that the combined DOR was 10.67 (95% CI = 3.73–30.53). In addition, the threshold effect analysis showed that the threshold effect was 0.23 and the correlation coefficient was −0.48, indicating that there was no threshold effect. In the forest map, the DOR of each study and the combined DOR are not distributed along the same line, and *Q* = 2.2 × 10^14^, *P* ≤ 0.001. Furthermore, the metaregression analysis of PCT study design, bacterial infection site, and mean age displayed that the *P* values were >0.05. The combined sensitivity was 0.77 (95% CI = 0.54–0.90), the combined specificity was 0.76 (95% CI = 0.70–0.82), the combined positive likelihood ratio was 3.25 (95% CI = 2.33–4.52), the combined negative likelihood ratio was 0.30 (95% CI = 0.14–0.67), and the combined AUC was 0.80 (95% CI = 0.76–0.83). In conclusion, PCT has moderate diagnostic value for adult liver failure complicated with bacterial infection, and it is a better auxiliary diagnostic index for liver failure with bacterial infection. However, the results of procalcitonin must be carefully interpreted combined with medical history, physical examination, and microbiological assessment.

## 1. Introduction

Liver failure is a kind of common end-stage liver disease in clinic with a high short-term mortality rate. It is caused by hepatitis B virus (HBV) and hepatitis C virus (HCV) or alcoholic hepatitis or hepatotoxic substances, etc., which leads to massive hepatocyte necrosis, cytokine storm, and systemic inflammatory response syndrome. In the short term, it seriously damages the physiological functions of liver. At the same time, liver failure is more susceptible to infection and increased levels of circulating proinflammatory cytokines and chemokines due to immune damage, abnormal bacterial translocation, local ischemia, and hypoxia. The levels of pathogen-associated molecular patterns (PAMPs) and the damage-associated molecular patterns (DAMPs) released by hepatocyte damage increased and led to systemic inflammatory response syndrome. Then, they can trigger immune-mediated tissue damage, produce higher levels of inflammatory cytokines and systemic markers of oxidative stress, lead to severe renal and hepatic failure, and exacerbate portal hypertension, hepatic encephalopathy, and death [1–10].

Among bacterial infections, spontaneous bacterial peritonitis (SBP) is the commonest type of infection followed by urinary tract infections and pneumonia [8, 11, 12]. Early diagnosis of all these infections and SBP is a critical step in the management of patients with liver failure. However, early clinical signs of bacterial infection in patients with liver failure, such as fever, tachycardia, leukopenia, hypotension, and thrombocytopenia, are not specific. In addition, some of them overlap with symptoms of liver failure, which can easily mask the condition and lead to delayed diagnosis and treatment, prolonged hospitalization, as well as increased mortality and costs [13, 14]. Since the presentation of any bacterial infection may not be typical, clinical suspicion is extremely significant. Although bacterial culture is the “gold standard” for the diagnosis of bacterial infections, its sensitivity is poor and it takes a long time (>24 hours), which is also too late for life-saving treatment. Consequently, it is essential to discover early, quick, and responsible diagnostic biomarkers of bacterial infections in patients with liver failure.

Bacterial infections can activate the cellular and humoral immune systems, releasing a variety of substances to mediate the host response to infection. Procalcitonin (PCT) is a 116 amino acid glycoprotein with a broad biological range, a short induction time after bacterial stimulation, a long half-life, and low concentrations in viral infections and nonspecific inflammatory diseases. It can be used to diagnose bacterial infection and to assess their severity and predict prognosis [15, 16].

With the continuous progress of understanding of PCT, there are many studies on the accuracy of PCT in the diagnosis of liver cirrhosis complicated with bacterial infection [17–19]. However, the value of using PCT levels for early detection of bacterial infections in patients with liver failure is controversial [20, 21]. Furthermore, there is still a lack of meta-analysis regarding the accuracy of PCT in the diagnosis of bacterial infections complicating liver failure. Therefore, in order to understand the accuracy of PCT in the diagnosis of adult liver failure complicated with bacterial infection, this study conducted a meta-analysis of the published literatures on the diagnostic value of PCT in adult liver failure complicated with bacterial infection and comprehensively and quantitatively evaluated its application value.

## 2. Materials and Methods

### 2.1. Literature Search Strategy

We conducted a comprehensive search of Medline, Embase, ISI Web of Knowledge, Cochrane Library, Scopus, and Science Direct for studies assessing the diagnostic accuracy of procalcitonin for bacterial infections in patients with liver failure. We scoured the databases from inception to March 28, 2021. Furthermore, we also manually searched the references that have been included in each primary study identified.

Our medical subject Mesh terms (for Medline), Emtree terms (for Embase), and text (for others) were “(procalcitonin or PCT) and (sepsis or “bacterial infection” or “systemic inflammatory response syndrome” or SIRS) and (“liver failure” or “hepatic failure” or “severe hepatitis” or “liver cirrhosis”)”. Studies were included if they evaluated the accuracy of procalcitonin for differentiation between liver failure patients with bacterial infection from those without infection.

### 2.2. Inclusion Criteria

(1) The aim of this study was to assess or explore the diagnostic value of PCT for bacterial infection in liver failure. (2) The subjects were adults over 18 years old. The experimental group was patients with liver failure complicated with infection, and the control group was patients with liver failure without infection. (3) Diagnostic criteria: bacterial pneumonia was defined as the association of clinical and radiological signs of lung infection observed in chest radiographs: fever, cough, cough sputum, imaging changes of pulmonary infection, positive qualified sputum culture. Spontaneous bacterial peritonitis was diagnosed when ascites culture was positive or ascites neutrophils greater than 0.25 × 10^9^/L, excluding other secondary inflammations such as cancer, tuberculosis, and rupture or perforation of abdominal organs. Urinary tract infection was clinically confirmed when the detection found more than 10 leukocytes per high power field in positive urinary culture or uncountable leukocytes per field in negative urinary culture. Patients with infection and SOFA score ≥ 2 were diagnosed with sepsis [8, 12]. (4) It can directly or indirectly obtain four values including true positive value, false positive value, true negative value, and false negative value of PCT in the diagnosis of adult liver failure with bacterial infection.

### 2.3. Exclusion Criteria

1. Animal experiments
2. Reviews, letters, case reports, comments, conference abstracts, and editorials
3. Subjects were healthy or uninfected patients, children under 18 years of age
4. The data are incomplete

### 2.4. Data Extraction and Literature Quality Evaluation

Two researchers independently extracted the data of the included literatures. Divergences were resolved in consensus sessions. In contrast, if agreement cannot be united, it is resolved by referral to a third investigator. We used the Quality Assessment of Diagnostic Accuracy Studies-2 (QUADAS-2) tool to evaluate the study quality and potential for bias assessment. Quality assessment is a general assessment of the quality of the included studies, which is useful for exploring heterogeneity.

### 2.5. Statistical Analysis

QUADAS-2 was performed using the Review Manager (RevMan) [computer program]. The summary receiver operating curve (SROC), the combined sensitivity, combined specificity, combined diagnostic odds ratio (DOR), combined positive likelihood ratio (PLR), combined negative likelihood ratio (NLR), and their 95% confidence interval (95% CI) were calculated. Subgroup analyses of age, cutoff of PCT, acute-on-chronic liver failure versus other types of liver failure, and sepsis versus other cites of bacterial infection studies were performed to examine their effects on the results. Deek's test was used to assess the publication bias of the included literatures. Analyses were performed using Stata software (version 16.0; College Station, TX). *P* values less than 0.05 were regarded as statistical significance.

## 3. Results

### 3.1. Literature Search Results

A total of 480 relevant literatures were retrieved. After reviewing the titles, abstracts, and full text, the literatures that did not meet the inclusion criteria were excluded, and six articles were finally included [20–25]. These studies included 432 liver failure patients without bacterial infection, with 466 (51.89%) confirmed patients with bacterial infection. In addition, the number of subjects in each study varied from 50 to 386. The threshold of PCT in the diagnosis of liver failure with bacterial infection was 0.48–1.62 *μ*g/mL. Furthermore, the sensitivity and specificity were 43%–96% and 63%–100%, respectively. The author, publication year, and other characteristics in the included studies were recorded and are summarized in Table 1.

### 3.2. Literature Quality Evaluation (Figure 1)

With regard to patient selection bias, two retrospective studies did not explicitly report that patients were consecutive. As for flow and time, three studies reported the patients did not receive the same reference standard. The results of the QUADAS-2 quality assessment of the six studies were shown graphically as the proportion of studies with low, high, or unclear risk of bias (Figure 1).

### 3.3. Meta-Analysis of Diagnostic Accuracy of PCT in Liver Failure Complicated with Bacterial Infection

Figure 2 represents a forest plot of the sensitivity and specificity of PCT assays used to diagnose bacterial infections in patients with liver failure in six studies. The sensitivity varied widely, from 0.43 to 0.96 (pooled 0.77, 95% confidence interval [CI] 0.54–0.90), while specificity ranged from 0.63 to 1.00 (pooled 0.76, 95% CI 0.70–0.82) (Figure 2). It was of note that the pooled PLR (positive likelihood ratio) was 3.25 (95% CI 2.33–4.52), the NLR (negative likelihood ratio) was 0.30 (95% CI 0.14–0.67), and the DOR (diagnostic odds ratio) was 10.67 (95% CI 3.73～30.53) (Table 2). The wise square values for sensitivity, specificity, PLR, NLR, and DOR were 94.85, 80.99, 77.81, 95.09, and 100.00, respectively. *P* values for sensitivity, specificity, PLR, NLR, and DOR were all 0.00, indicating remarkable heterogeneity among studies in terms of sensitivity, specificity, PLR, NLR, and DOR.

To compare average age over 50 years old studies with below 50 years old (three provided data for average age over 50 years old patients and three provided data for below 50 years old patients), the level of cutoff over 1 *μ*g/mL studies with below 1 *μ*g/mL (two provided data for the level of cutoff over 1 *μ*g/mL patients and four provided data for below 1 *μ*g/ml patients), acute-on-chronic liver failure studies with other types of liver failure studies (four provided data for acute-on-chronic liver failure patients and one provided data for chronic severe hepatitis patients and one provided data for acute liver failure patients), sepsis with other sites of infection (one provided data for spontaneous bacterial peritonitis patients, two provided data for sepsis patients, and three provided data for other sites of bacterial infection patients), we did a subgroup analysis. Analysis of these variates yielded no significant results (Table 3). Hence, these factors could not explain the heterogeneity among the studies.

### 3.4. Publication Bias

The potential publication bias of the meta-analysis was analyzed using Deek's test. The test showed *P*=0.08, demonstrating that there was no publication bias in our studies.

## 4. Discussion

Bacterial infection has been acknowledged as a potential trigger factor in a fair number of complications of end-stage liver disease with hepatic encephalopathy, renal failure, and coagulation disorders; deterioration of liver function; and even death. Early recognition of bacterial infection is difficult because of the absence of typical clinical manifestations in this patient population. At present, bacterial culture is the “gold standard” for the diagnosis of bacterial infection while the sensitivity is poor, and it takes a long time (>24 h). Most time, the early diagnosis of bacterial infection requires clinicians to confirm by their careful medical history, physical examination, radiological examination, microbiological examination, and dynamic observation of disease changes. However, due to the varying experience of doctors or the complexity of the disease, the clinical diagnosis is difficult to make. Therefore, it is necessary that a rapid and accurate laboratory biomarker can be used to assist diagnosis and treatment, thereby reducing the risk of death, antibiotic abuse, and the risk of antibiotic-related side effects. In short, PCT detection is easy to be operated and obtained quickly.

PCT production mainly comes from the liver, and the concentration was almost undetectable during endotoxin shock when the liver was resected [26]. Theoretically, liver disease should affect PCT synthesis and its production concentration in the blood should be negatively correlated with the severity of liver disease. Conversely, some studies have revealed that the concentration of PCT can predict hepatocellular damage and the more serious the liver disease, the higher the procalcitonin level [27–30]. The reasons for the increase of procalcitonin concentration may be on the one hand, the intestinal barrier of patients with liver cirrhosis or liver failure was damaged, and the intestinal bacteria were ectopic, which led to endotoxemia and the increase of PCT synthesis; on the other hand, the damage, apoptosis, or necrosis of hepatocytes resulted in the release of damage-associated molecular patterns (DAMPS), activated the downstream pathways including IL-1*β* and TNF-*α*, and stimulated the expression of PCT [16, 31]. Although the level of PCT was associated with liver damage, more and more studies have found that procalcitonin still has certain guiding significance for liver disease patients with bacterial infection. Bota et al. [32] suggested that bacterial infected patients with liver cirrhosis had the same concentrations of PCT and CRP as those without cirrhosis. Procalcitonin serum levels can help identify infected patients with alcoholic hepatitis [27, 33, 34] and are better than CRP in distinguishing between the cause of infection and systemic inflammatory response [18, 33, 34]. Unfortunately, there is a lack of systematic research and evaluation on its diagnostic accuracy.

Based on the results of six studies, we obtained that the pooled sensitivity, specificity, DOR, and AUC of PCT were 0.77, 0.76, 10.67, and 0.80, respectively, indicating that procalcitonin is of medium diagnostic value in distinguishing bacterial infection from nonbacterial infection in patients with liver failure.

Combined likelihood ratios can distinguish the ability of diagnosis of disease (sensitivity) and nondisease (specificity), which has important clinical significance. In our study, both positive likelihood ratio and negative likelihood ratio were moderate (Figure 3). A positive likelihood ratio of 3 means that the probability of PCT positive in patients with bacterial infection is three times that in patients without bacterial infection, which means that patients with high serum procalcitonin concentration are more likely to consider bacterial infection than patients with low serum procalcitonin concentration. By comparison, our study found a negative likelihood ratio of 0.30, which means that if the PCT test result is negative, the possibility of bacterial infection is 7%, whereas plasma procalcitonin concentration is related to the degree of liver injury and infection. Likelihood ratios are calculated from binary variables and partly distorted, so it cannot be used as a tool to rule-in and rule-out bacterial infection. Moreover, the results of procalcitonin assay should be interpreted in the context of a detailed history, physical examination, and microbiological findings.

In our study, there are still some limitations. We observed a considerable heterogeneity. Then, we found that the mean age, type of liver failure, infection site, and PCT threshold were not responsible for the heterogeneity. Our heterogeneity may be mainly related to the following aspects: firstly, differences in the etiology of liver disease and severity of liver function in different studies may be a source of heterogeneity. Nonetheless, due to the lack of specific conditions of each patient in each study and the limited number of articles meeting our inclusion criteria, it not only hindered the metaregression analysis but also affected our more specific subgroup analysis. Thus, it is hard to discover the origin of heterogeneity. Secondly, the cutoff of PCT differed between studies, leading to the difference of sensitivity and specificity of different studies. Thirdly, because of the absence of detailed records in the initial paper, we cannot evaluate the impact of PCT testing technology, laboratory infrastructure, and settings on the accuracy of PCT measurement. In addition, the low-quality evaluation we have included in the study may generate overestimation of the accuracy of diagnosis. Meta-analysis has been a widely used tool in the analysis of clinical cases [35, 36]. Along with other mathematical tools [37, 38], comprehensive medical analysis can be achieved in future works according to the methods and findings of this paper.

## 5. Conclusions

In summary, procalcitonin is a useful marker for the diagnosis of bacterial infection in patients with liver failure. However, bacterial infection is a pathophysiological process rather than a specific syndrome, and it is so complicated that it cannot be assessed by a single measurement. Clinicians should combine detailed medical history, physical examination, radiology examination, microbiology examination, and other comprehensive judgment to explain and monitor the changes of procalcitonin levels dynamically. At the same time, due to the limitations of the conclusions of this study, we look forward to more studies with larger sample size, especially high-quality large-scale randomized controlled trials involving different regions and races.

## Figures and Tables

**Figure 1:** Methodological evaluation of the included studies according to QUADAS-2. Graphical display of the QUADAS-2 results showing the proportion of studies with high, low, or unclear risk levels of bias. QUADAS-2 = Quality Assessment of Diagnostic Accuracy Studies-2.

**Figure 2:** Forest plot of estimates of sensitivity and specificity for procalcitonin assays in the diagnosis of bacterial infection in liver failure patients. The point estimates of sensitivity and specificity from each study are shown as solid circles. Error bars indicate 95% CIs. CI = confidence interval.

**Figure 3:** Fagan nomogram of the procalcitonin test for diagnosis of bacterial infection in liver failure patients.

**Table 1:** Characteristics of the six included studies.

Author	Year	Mean age (year)	Etiology	Diagnosis of liver failure	Site of infection	Cutoff (ng/mL)	*n*	Prevalence (%)	TP	FP	FN	TN	Sensitivity (95% CI)	Specificity (95% CI)
Yuan et al.	2013	56	Chronic severe hepatitis B	PTA < 40%	Sepsis	0.48	84	50	16	6	8	51	0.95 [0.84–0.99]	0.79 [0.63–0.90]
Rule et al.	2015	41	Acute liver failure	PT > 15 seconds or INR ≥ 1.5 IU + HE within 26 weeks	Sepsis	1.62	115	49	87	8	7	27	0.64 [0.50–0.77]	0.63 [0.49–0.75]
Qu et al.	2016	44	ACLF	TB ≥ 5 mg/dL + INR ≥ 1.5 + ascites and/or HE within 4 weeks	Bacterial infection	0.61	120	57	65	15	3	37	0.96 [0.88–0.99]	0.71 [0.57–0.83]
Zhang et al.	2018	59	ACLF	EASL criteria		0.57	50	74	27	0	10	13	0.73 [0.56–0.86]	1.00 [0.75–1.00]
Chen et al.	2020	47	ACLF	TB ≥ 5 mg/dL + INR ≥ 1.5 + ascites and/or HE within 4 weeks	Sepsis	0.765	143	66	52	9	42	40	0.55 [0.45–0.66]	0.82 [0.68–0.91]
Lin et al.	2020	52	ACLF	TB ≥ 5 mg/dL + INR ≥ 1.5 + ascites and/or HE within 4 weeks		1.01	386	44	72	46	97	171	0.43 [0.35–0.50]	0.79 [0.73–0.84]

HE: hepatic encephalopathy; TB: total bilirubin; ACLF: acute-on-chronic liver failure; EASL criteria: (1) patients with single kidney failure, (2) patients with single failure of the liver, coagulation, circulation, or respiration who had a serum creatinine level ranging from 1.5 to 1.9 mg/dL and/or mild to moderate hepatic encephalopathy, and (3) patients with single cerebral failure who had a serum creatinine level ranging from 1.5 to 1.9 mg/dL.

**Table 2:** Meta-analysis results derived from the 2 × 2 tables of individual studies using serum procalcitonin as a marker for bacterial infection in liver failure patients.

Author	Year	DOR (95% CI)	PLR (95% CI)	NLR (95% CI)
Yuan et al.	[22]	73.33 (14.81–363.22)	4.44 (2.48–7.96)	0.06 (0.02–0.24)
Rule et al.	[20]	3.03 (1.42–6.47)	1.72 (1.17–2.53)	0.57 (0.38–0.85)
Qu et al.	[23]	53.44 (14.51–196.82)	3.31 (2.16–5.09)	0.06 (0.02–0.19)
Zhang et al.	[24]	70.71 (3.85–1000.00)	20.26 (1.32–310.36)	0.29 (0.17–0.48)
Chen et al.	[25]	5.50 (2.40–12.61)	3.01 (1.62–5.59)	0.55 (0.42–0.71)
Lin et al.	[21]	2.76 (1.77–4.31)	2.01 (1.47–2.74)	0.73 (0.63–0.84)
Overall		10.67 (4.07–25.33)	3.25 (2.33–4.52)	0.30 (0.14–0.67)
*I* ^2^		100.00 (100.00–100.00)	77.81 (77.81–96.00)	95.09 (92.52–97.66)

**Table 3:** Meta-analysis results derived from subgroup analysis using serum procalcitonin as a marker for bacterial infection in liver failure patients.

Subgroup	*P* value	*I* ^2^ (%)
Age, more than 50 years old	≤0.001	89.5
Age, less than 50 years old	≤0.001	85.7
Etiology, ACLF	≤0.001	86.4
Etiology, nACLF	≤0.001	92.0
Site, sepsis	0.002	83.9
Site, nsepsis	≤0.001	90.7
Cutoff, more than 1 *µ*g/mL	0.837	0.0
Cutoff, less than 1 *µ*g/mL	0.003	78.8

ACLF: acute-on-chronic liver failure; nACLF: non-acute-on-chronic liver failure; nsepsis: non-sepsis.

## Data Availability

All data supporting this meta-analysis are from previously reported studies and data sets, which have been cited. The processed data are available at Medline, Embase, ISI Web of Knowledge, Cochrane Library, Scopus, and Science Direct, from inception to Mar 28, 2021.
